# Downregulated Poly-C binding protein-1 is a novel predictor associated with poor prognosis in Acute Myeloid Leukemia

This article has been retracted.

**DOI:** 10.1186/s13000-015-0377-y

**Published:** 2015-08-21

**Authors:** Meifeng Zhou, Xiuzhen Tong

**Affiliations:** Department of Hematology, the First Affiliated Hospital of Sun Yat-sen University, Guangzhou, Guangdong 510080 China

## Abstract

**Background:**

Depletion of Poly-C binding protein-1(PCBP1) is implicated in various human malignancies. However, the underlying biological effect of PCBP1 in cancers, including acute myeloid leukemia (AML), still remains elusive. The purpose of this study was to examine the expression and clinical outcome of PCBP1in acute myeloid leukemia.

**Methods:**

Bone marrow fluids of 88 newly diagnosed AML patients were sampled, and the PCBP1 mRNA expression level was evaluated using quantitative RT-PCR. The association between PCBP1 expression and clinicopathological features or the survival status of the patients was assessed by Chi-square test and Kaplan-Meier method.

**Results:**

Comparing newly diagnosed AML patients to normal healthy donors, PCBP1 expression was significantly decreased in AML patients (P < 0.001). Conversely, PCBP1 expression had accordingly recovered back to normal in patients with complete remission (P < 0.001). Clinical feature analyses showed that PCBP1 expression was negatively correlated with white blood cell count (P = 0.024). In addition, patients with low PCBP1 expression had poor disease-free survival (11.8 % vs. 45.3 %; P = 0.01) and overall survival (18.2 % vs. 42.4 %; P = 0.032), respectively.

**Conclusions:**

Taken together, our results showed for the first time that expression of PCBP1 was down-regulated in newly diagnosed AML patients and might be an independent prognostic marker in AML and should to be further investigated.

## Background

Acute myeloid leukemia (AML) is a clinically and genetically heterogeneous disease characterized by the differentiation arrest and the malignant clonal proliferation of hematopoietic progenitor cells [1, 2]. It is the most common myeloid leukemia and accounts for 70 % of acute leukemia in adults [3–5]. Exposure to ionizing radiation, benzene, and cytotoxic chemotherapy is known to increase the incidence of AML [3]. The pathogenesis of AML is highly complex. Over the past decades, researching in genetic alterations, such as FLT3, NPM1, CEBPA gene mutations, resulted in prodigious improvement in the pathogenesis, prognostic classification and novel therapeutic approaches of AML [6, 7]. Despite the noteworthy progress in the development of genomic studies on AML, the prognosis classification and treatment for most AML patients still remains unsatisfactory [7–10]. More than half of young adult patients and about 90 % of elder patients still die of the disease, due to either resistance to therapy or relapsed AML, and the 5-year survival rate is less than 30 % [11–13]. As a result, more effective gene signatures are still required for risk-adapted treatment [14]. In addition, clinical outcomes can differ greatly in patients with identical karyotypes, suggesting that additional factors on AML diagnosis and prognosis should be identified and clarified [12]. Thus, investigation for more valuable diagnostic, prognostic factors and therapeutic targets implicated in AML pathogenesis is pressing for the performance of individual antitumor treatment.

Poly-C binding protein 1, also referred to as hnRNP-E1 or αCP-1 [15], is broadly expressed in many human tissues and organs, including bone marrow, as well as the liver, heart, kidneys, brain, lungs, and placenta. Functionally, PCBP1 is known to play multiple roles in a wide spectrum of transcriptional and posttranscriptional events, including in mRNA transcription regulation, transportation, splicing, translation, and stabilization by means of its cis-DNA/RNA-binding activity [16–18]. Increasing clinical and cellular evidence has demonstrated that PCBP1 plays pivotal roles in multiple pathological processes, including cancer apoptosis, metastasis, invasion and malignant transformation [17, 19–21]. Recently, some studies indicated that aberrant expression of PCBP1 is associated with poor prognosis [22], and low PCBP1 expression could be a poor prognosis marker in diverse human cancers [17, 23].

Although aberrant PCBP1 expression levels are associated with cancer progression and metastases in many human solid cancers, there is not a straightforward experiment to demonstrate this role in tumor formation. Likewise, the function of PCBP1 in leukemia, including AML remains elusive. Herein, our study was carried out to investigate PCBP1 expression in AML and to understand the prognostic role of PCBP1 in AML patients.

## Methods

### Patients and tissue samples

A myeloid neoplasm with 20 % or more myeloblasts in the peripheral blood or bone marrow is considered to be AML according to the 2008 World Health Organization (WHO) criteria [24]. Initial diagnosis of AML samples prior to AML treatment were collected as newly diagnosed of acute myeloid leukemia. 88 patients, who were newly diagnosed with AML, were admitted for treatment at the First Affiliated Hospital of Sun Yat-sen University from 2012 to 2015. All patients underwent a bone marrow puncture at the time of diagnosis, with a signed informed consent. Morphology, Immunology, Cytogenetics and Molecular Biology (MICM) classification was performed on the bone marrow. Clinical features of all patients were summarized in Table 1, and the risk status was predicted on the basis of validated cytogenetics and molecular abnormalities. According to NCCN guidelines version 2.2013, we classified acute myeloid leukemia risk-status into three categories: better-risk (inv(16),t(16;16),t(8;21),t(15;17) or NPM1 mutation in the absence of FLT3-ITD with normal cytogenetics), poor-risk (complex monosomal karyotype, −5, 5q-,-7,7q-,11q23 abnormality, inv(3), t(3;3), t(6;9), t(9;22) or normal cytogenetics with FLT3-ITD mutation) or intermediate-risk (neither better-risk nor poor-risk). Meanwhile, 24 healthy donors were recruited as normal control with their permission. Complete remission (CR) was defined by the presence of all the following: less than 5 % myeloid blasts in bone marrow, no leukemic blasts in peripheral blood, absolute neutrophil counts ≥ 1,500/μl and platelet counts ≥ 100,000/μl in peripheral blood, and no persistence of extramedullary disease [25]. The clinical characteristics of these newly diagnosed patients were listed in Table 1. Sixty-seven patients were further followed up. In analysis of the disease-free survival, data were censored at the time of relapse, death or the last contact; in analysis of the overall survival, data were censored when the patients died or last known to be alive. This study was approved by the local ethic committee of the First Affiliated Hospital of Sun Yat-sen University and informed consents were obtained from each patient.

**Table 1:** Characteristics of AML patients in this study

Variables	No. of patients (%)
Age, (range, year old)	41 (14-79)
Sex ration, male/female	61/27
Median wbc, ×10^9^/L,(range)	24.96 (0.85-395)
Blast cell in bone marrow, % (range)	56 (20-96)
FAB category:	
M0/M1	8 (9.09 %)
M2	19(21.59 %)
M3	11(12.5 %)
M4/M5	44(50.0 %)
M6/M7	6(6.82 %)
Risk status:	
Better-risk	21(23.86 %)
Intermediate-risk	44(50.0 %)
Poor-risk	23(26.14 %)

### Preparation of mononuclear cells and RNA extraction

Bone marrow fluid from each patient was obtained using a 6-ml EDTA-containing vacutainer. The collected sample was then diluted with physiological saline in 1:1 proportion, the diluted sample was carefully layered over the ficoll lymphocyte separation medium (LSM, MP Biomedicals, USA) and centrifuged at a speed of 400 × g at room temperature for 20 minutes. During centrifugation, differential migration results in the formation of four cell layers: plasma layer, mononuclear cell layer, LSM layer and RBC pellet. Erythrocytes and polynuclear leukocytes sedimented to the bottom of the tube; mononuclear cells were found at the plasma-LSM interface. After aspirating the mononuclear cells and transferring them to a new centrifuge tube, cells were washed twice with buffered balanced salt solution and re-suspended in 1 ml TRIzol reagent (Cwbio Cat: CW0580A). Total cellular RNAs were then extracted according to the guideline of the Ultrapure RNA Kit (Cwbio Cat: CW0581, China) and eluted in 30–50 μl of RNase-free water. The RNA concentration and quality were determined by NanoDrop 1000 spectrophotometer (ThermoFisher Scientific, USA).

### Reverse transcription

To obtain cDNA, 2 μg of total RNA were diluted into nuclease-free water to a total volume of 12 μl, mixed with 1 μl of anchored-oligo (dT) 18 primer (2.5 μM) and incubated for 10 minutes at 65 °C to denature the template-primer mixture. After that, the remaining components of the RT mix, 4 μl transcriptor RT reaction buffer (5×), 0.5 μl protector RNase inhibitor (40 U/ul), 2 μl deoxynucleotide Mix (10 mM) and 0.5 μl transcriptor reverse transcriptase (20 U/μl) were added to the tube. The 20 μl reaction volumes were incubated at 55 °C for 30 minutes followed by 5 minutes at 85 °C, and the reaction was then halted by placing the tube on ice. All cDNAs were diluted to 1:10 in nuclease-free water and stored at -20 °C for use.

### Quantitative real-time PCR analysis for PCBP1 expression

In order to quantify PCBP1 mRNA expression levels, primers 5’-CATCCGCTAAGAATTTAAAAAT-3’ (forward) and 5’-AAGACAGCAATTCCCAGC-3’ (reverse) were used. Meanwhile 5’-ACCACAGTCCATGCCATCAC-3’ (forward) and 5’-TCCACCACCCTGTTGCTGTA-3’ (reverse) were used for amplification of the internal control gene GAPDH. Quantitative real-time PCR (qRT-PCR) were performed according to the instructions of RealMasterMix (SYBR Green) kit (Tiangen Biotech, China). Briefly, in each total volume of 20 μl reaction mixture, 9 μl of 2.5 × RealMasterMix/20 × SYBR Solution, 0.4 μl of forward and reverse primers(10 μM), 2 μl of diluted cDNA and 8.2 μl of ultrapure water were added. Amplification was conducted on a CFX96 Real-time fluorescent quantitative PCR detection system (Bio-Rad, USA) with the thermal cycling parameters as the initial denaturation at 95 °C for 2 minutes, following by 40 cycles of 20 seconds at 95 °C, 30 seconds at 60 °C, 40 seconds at 68 °C. Melting curves were drawn to identify the specificity of the PCR primers. Each experiment was repeated at least for three times.

Relative quantification of PCBP1 expression was calculated by the comparative cycle threshold method (the 2^-ΔΔCT^ method) [26], where ΔΔCT = ΔC_T,Target_ - ΔC_T,Control_. The change in expression of PCBP1 was normalized to its internal control GAPDH, just as ΔC_T,Target_ = C_T,Target_ - C_T,GAPDH_. Meanwhile, the smallest numeric values of 2^-ΔCT, Target^ was defined as “1” as a control; the relative PCBP1 mRNA expression of other AML sample, CR patients and healthy donors were carried out by folds of the control.

### Statistical analysis

Statistical analysis was performed by SPSS12.0 statistical software. The data was expressed as the mean ± standard deviation (SD) or mean ± SEM of at least 3 independent experiments. The Student T test was used to compare continuous variables. Different frequencies between groups were compared by the chi-square test or the Fisher exact test. Survival curves were obtained by the Kaplan-Meier method, and differences in survival among groups were analyzed by the log-rank test. P values < 0.05 were considered statistically significant.

## Results

### PCBP1 was significantly down-regulated in newly diagnosed AML patients

In order to explore whether PCBP1 is aberrantly expressed in AML patients, total RNA was isolated from bone marrows of AML patients and healthy donors, and the relative expression level of PCBP1 was detected using quantitative RT-PCR (qRT-PCR). The averaged relative value of PCBP1expression in newly diagnosed AML patients (averaged expression value 7.08, n = 88) was significantly lower than that in normal controls (averaged expression value 19.31, n = 24) (Fig. 1, P < 0.001). Furthermore, among 12 patients who achieved CR after one or two cycles of chemotherapy, PCBP1 expression level had markedly recovered back to their initial admission level (mean, 20.96 versus 6.25) (Fig. 2, P < 0.001), although it was higher than that of the normal controls, there was no statistical difference (mean 20.96 versus 19.31, p > 0.05) (Fig. 3). Therefore, the results revealed that PCBP1 expression level in the majority of AML patients was negatively related to the state of the illness of AML.

**Fig. 1:** PCBP1 was down-regulated in AML patients.The relative PCBP1 mRNA expression in newly diagnosed AML patients (n = 88) and healthy donors (n = 24) by qRT-PCR evaluation. PCBP1 expression was significantly decreased in newly diagnosed AML patients (average 7.08) compared with healthy donors (average 19.31; P < 0.001). Each experiment was performed at least in triplicate

**Fig. 2:** Comparison of PCBP1mRNA expression in 12 newly diagnosed/complete remission paired samples. Comparison of PCBP1 mRNA expression of patients in complete remission (CR) with their initially diagnosed counterparts.PCBP1 expression in patients achieved CR is 20.96 ± 3.22 versus 6.25 ± 1.72; paired t test, P < 0.001

**Fig. 3:** Comparison of PCBP1 expression level in CR patients with normal controls.Comparison of PCBP1 expression in CR patients with that in healthy donors.CR, 20.96 ± 3.22 versus donors, 19.31 ± 3.3, P > 0.05

### Low PCBP1 expression was associated with advanced AML clinical characteristics

To question the relationship of PCBP1 expression to AML characteristics, the 88 AML patients were classified into two groups according to the averaged PCBP1 expression, in which patients with PCBP1 expression value less than their averaged level (7.08) were classified into low-expression group (mean expression value 3.12, n = 63), whereas patients with equal PCBP1 level or above the mean value were assigned to the high-expression group (mean expression value 17.06, n = 25), of them, 71.6 % (63/88) patients showed low PCBP1 expression. PCBP1 expression and clinical features were summarized in Table 2. The white blood cell count greater than or equal to 50 × 10^9^/L was identified in 30 (34.1 %) of 88 patients with AML and the frequency of PCBP1 underexpression was 86.7 % (26/30) in this subtype, whereas in 58 (65.9 %) AML patients with leukocyte count less than 50 × 10^9^/L, only 63.8 % (37/58) cases showed low-pcbp1 expression. Univariant analysis demonstrated that low PCBP1 expression was individually associated with high white blood cell count (P = 0.024). However, there was no significant correlation of PCBP1 expression with other clinical risk-predicting factors including FAB category (P = 0.413), risk status (P = 0.143), CD7 expression (P = 0.343), and CD56 expression (P = 0.563) (Shown in Table 2), indicating PCBP1 could be an independent prognostic marker.

**Table 2:** Association of PCBP1 expression to clinical features

			PCBP1 Expression		
Variables	Cases	Sum	Low	High	P
Age	<60	76	54	22	1.0
	≥60	12	9	3	
Sex	Male	61	44	17	0.866
	Female	27	19	8	
WBC	<50×10^9^/L	58	37	21	0.024^*^
	≥50×10^9^/L	30	26	4	
Blast in BM	<50 %	38	28	10	0.704
	≥50 %	50	35	15	
FAB category	M4/M5	44	33	11	0.413
	M1/M2	23	14	9	
	Others	21	16	5	
Risk status	Better	21	13	8	0.143
	Intermediate	44	30	14	
	poor	23	20	3	
CD56	positive	25	19	6	0.563
	negative	63	44	19	
CD7	positive	20	16	4	0.343
	negative	68	47	21	

^*^P < 0.05

### Association of PCBP1 expression to survival of AML patients

To further investigate the prognostic value of PCBP1 expression in patients with AML, sixty-seven CR patients with non-M3 acute myeloid leukemia were followed up. The effect of PCBP1 expression on non-M3 AML patients’ survival time was assessed by the Kaplan-Meier method with the log-rank test. Results revealed that the low-PCBP1 expression group had a clearly poor disease-free survival (11.8 % vs. 45.3 %; log rank P = 0.01; shown in Fig. 4a) and overall survival (18.2 % vs. 42.4 %; log rank P = 0.032; shown in Fig. 4b), confirming that PCBP1 could be an additional predictor in AML prognosis.

**Fig. 4:** Kaplan-Meier curves of DFS and OS. The Kaplan-Meier survival analysis of the DFS (**a**) and OS (**b**) in 67 newly diagnosed non-M3 AML patients with CR. High PCBP1 group, n = 23; Low PCBP1 group, n = 44, p < 0.05

## Discussion

Poly(C)-binding proteins (PCBPs), which are also well known as the heterogeneous nuclear ribonucleoprotein (hnRNP) family, were initially defined by their sequence-specific binding ability to polycytosine [poly (C)] in protein-nucleic acids interaction. In recent years, accumulating evidence has shown that PCBPs play a critical role in tumor development and progression [27,28]. Among PCBPs, hnRNP K, PCBP1, and PCBP2 have been intensively studied. HnRNP K, which is overexpressed in diverse neoplasms [29], can activate the transcriptional activation of oncogenes c-SRC and c-Myc [30,31], hinting its cancer-promoting potential. Upregulation of PCBP2 was also shown in the higher grades of human glioma [32] and PCBP2 can facilitate gastric cancer growth by targeting miR-34a [33]. More and more observations have described that PCBP1 could be implicated in malignancies [16, 23, 31] via in vitro cell line analyses and clinical observations. Mechanistically, PCBP1 silence facilitated androgen receptor (AR) protein expression by binding to the 3’ untranslated region (UTR) of AR mRNA in prostate cancer LNCap cells [34]. The phosphorylated PCBP1 mediated by TGF β signaling could promote epithelial-mesenchymal transition [35]. Accordingly, silencing endogenous PCBP1 in human SH-SY5Y cells resulted in a large body of altered transcripts, of which some are involved in Wnt signaling and TGF beta signaling [36]. NF-Kappa B pathway is also implicated in cancer metastasis, relapse and drug resistance, and PCBP1 is shown to inhibit NF-Kappa B activity by interacting with STAT3 pathway in HEK293 cells [37]. Furthermore, the other advances on the biological function and molecular mechanisms of PCBP1 involving in gene regulation were graphically represented in Fig. 5 [38]. Recent data disclosed that PCBP1 modulated P63 expression via mRNA stability [39]. Our previous results also demonstrated that PCBP1 downregulates metastatic PRL-3 phosphatase translation by interacting with its 5’ UTR [17].

**Fig. 5:** Schematic representation of signaling network involving PCBP1. Adapted from Ref. [38]

It has also been demonstrated that aberrant expression of PCBP1 promotes tumor development and progression [19]. Recent studies have revealed PCBP1 could increase the expression of P21^WAF1^ to reduce cell proliferation and tumor growth and play as a tumor suppressor in human solid cancer [17, 40]. In addition, our previous study had clearly demonstrated that PCBP1 repressed metastatic PRL-3 translation, resulting in the decreased tumorigenic ability of tumor cells [17]. Interestingly, PRL-3 has been reported to be upregulated in de noveo FLT3-ITD-negative AML patients [41] and involved in AML leukemogenesis [41] [42], indicating PCBP1 as a tumorsuppressor gene in AML progression. Our data is comparable with above reports and found that PCBP1 expression in newly diagnosed AML is obviously lower than that observed in healthy control donors. The results are also well consistent with observations that PCBP1 expressions are usually downregulated in some human tumors, including liver [19], gall bladder [23], choriocarcinoma [22], colon and lung cancers [17], as well as in metastatic cervical cancer [21] and metastatic breast cancer cells [43].Then, we found that the expression of PCBP1 in 12 AML patients in complete remission after intensive chemotherapy was also markedly increased, compared to that at their initial diagnosis, suggesting the dysregulated expression of PCBP1 is consistent with cancer progression. Similar results are also reported in other studies, such as Pillai MR et al. reported that reduced PCBP1 expressed in higher grade squamous intraepithelial lesions of cervical tissues and even progressed to cervical cancer [21].In addition, we analyzed the clinicopathological factors of PCBP1 in AML. Our results showed that low level of PCBP1 expression is positively correlated with the high counts of white cells, which represented more aggressive clinical features. The difference in other aggressive clinical features, including age, risk status and leukemic blasts, was not significant. Moreover, when compared to the patients with high PCBP1 expression, low PCBP1 expression AML patients have poorer overall and disease-free survival rates, indicating that PCBP1 expression can be considered as a novel prognostic marker in initial diagnosis of AML. Given that PCBP1 is involved in gene regulation through multiple roles, including transcription, translation and mRNA stabilization. PCBP1 should possibly participate in the blockade of tumorigenesis by either inhibiting particular oncogene expression or enhancing tumor suppressor expression in AML progression. Whatever, the detailed underlying mechanism of PCBP1 in AML progression will be further investigated and a potent novel target could be dug out in the PCBP1-silencing tumors.

To the best of our knowledge, the current study is the first to demonstrate that PCBP1 is downregulated in AML patients and accounts for approximately 72 % of newly diagnosed AML patients compared to healthy donors. In this study, we screened PCBP1 expression and defined the average expression level of AML patients as a cutoff point to classify the patients into 2 groups, of them, 71.6 % (63/88) patients showed low PCBP1 expression. Similar work for confirming this novel gene was carried out in lung and colon carcinoma [17]. In that study, IHC analysis revealed that PCBP1protein expression is negative in 85.7 % (54/63) lung cancer tissue arrays and 91.7 % (66/72) colon cancer tissue arrays and the different expression level may be due to different cancer types. Furthermore, the real risk changes of PCBP1 downregulation in AML need to be further investigated.

## Conclusion

This study showed that PCBP1 was downregulated in newly diagnosed acute myeloid leukemia, and the decreased PCBP1 expression level was associated with adverse prognosis in AML. Our findings are well consistent with observations that PCBP1 expression was usually downregulated in a variety of solid tumors. However, the underlying molecular mechanism for PCBP1 in AML progression is not well elucidated and further investigation will be required.

## Abbreviations

AML: Acute myeloid leukemia
PCBP1: Poly-C binding protein-1
CR: Complete remission
DFS: Disease-free survival
OS: Overall survival
HnRNPs: Heterogeneous nuclear ribonucleoproteins
PCBPs: Poly(C)-binding proteins
